The article "EEG signature of grouping strategies in numerosity perception" was published in 2023. Journal: Front Neurosci.

# EEG signature of grouping strategies in numerosity perception

**DOI:** 10.3389/fnins.2023.1190317

**Published:** 2023-05-24

**Authors:** Camilla Caponi, Paula A. Maldonado Moscoso, Elisa Castaldi, Roberto Arrighi, Paolo A. Grasso

**Affiliations:** ^1^Department of Neuroscience, Psychology, Pharmacology and Child Health, University of Florence, Florence, Tuscany, Italy; ^2^Centre for Mind/Brain Sciences – CIMeC, University of Trento, Rovereto, Italy; ^3^Department of Physics and Astronomy, University of Florence, Florence, Tuscany, Italy

**Keywords:** groupitizing, subitizing, numerosity perception, EEG, ERPs

## Abstract

The moment we see a group of objects, we can appreciate its numerosity. Our numerical estimates can be imprecise for large sets (>4 items), but they become much faster and more accurate if items are clustered into groups compared to when they are randomly displaced. This phenomenon, termed groupitizing, is thought to leverage on the capacity to quickly identify groups from 1 to 4 items (subitizing) within larger sets, however evidence in support for this hypothesis is scarce. The present study searched for an electrophysiological signature of subitizing while participants estimated grouped numerosities exceeding this range by measuring event-related potential (ERP) responses to visual arrays of different numerosities and spatial configurations. The EEG signal was recorded while 22 participants performed a numerosity estimation task on arrays with numerosities in the subitizing (3 or 4) or estimation (6 or 8) ranges. In the latter case, items could be spatially arranged into subgroups (3 or 4) or randomly scattered. In both ranges, we observed a decrease in N1 peak latency as the number of items increased. Importantly, when items were arranged to form subgroups, we showed that the N1 peak latency reflected both changes in total numerosity and changes in the number of subgroups. However, this result was mainly driven by the number of subgroups to suggest that clustered elements might trigger the recruitment of the subitizing system at a relatively early stage. At a later stage, we found that P2p was mostly modulated by the total numerosity in the set, with much less sensitivity for the number of subgroups these might be segregated in. Overall, this experiment suggests that the N1 component is sensitive to both local and global parcelling of elements in a scene suggesting that it could be crucially involved in the emergence of the groupitizing advantage. On the other hand, the later P2p component seems to be much more bounded to the global aspects of the scene coding the total number of elements while being mostly blind to the number of subgroups in which elements are parsed.

The article "EEG signature of grouping strategies in numerosity perception" was published in 2023. Journal: Front Neurosci.

## Introduction

Humans share with other animal species the ability to produce rapid but approximate estimates of the number of elements in a set (Dehaene, 2011). This ability, based on the number sense, is thought to be hard wired in our perceptual system for a series of reasons: it is universal (Ferrigno et al., 2017), it is spontaneous (Cicchini et al., 2016, 2019; Castaldi et al., 2018, 2021), it is susceptible to adaptation (Burr and Ross, 2008; Arrighi et al., 2014; Castaldi et al., 2016; Grasso et al., 2021a,b), it is tuned to salient features (Grasso et al., 2022a) and it is evident from a few hours after birth (Izard et al., 2009; Anobile et al., 2021b).

Previous behavioural studies have identified two independent systems supporting numerosity perception: the *subitizing* system allowing rapid and errorless judgments of few elements (up to four; Jevons, 1871; Kaufman et al., 1949; Atkinson et al., 1976) and the *Approximate Number System* (ANS), a slower and less accurate system for larger sets of items (Dehaene, 2011). Interestingly, recent evidence showed that the precision of numerical estimates in the *estimation* range (i.e., the range of numerosities above subitizing) improved when grouping cues (allowing to parse the whole set into subgroups of few elements) are available, a phenomenon termed “groupitizing” (Starkey and McCandliss, 2014). Specifically, enumeration of quantities within the estimation range is faster and more precise when items can be grouped into clusters, provided the number of clusters and elements in each group falls within the subitizing range (Anobile et al., 2020; Ciccione and Dehaene, 2020; Maldonado Moscoso et al., 2020).

One of the hypothesis put forward to account for the groupitizing effect, posits it might rely on the recruitment of the subitizing system and calculation abilities (Anobile et al., 2020; Ciccione and Dehaene, 2020). Indeed, while adults can leverage on several grouping cues (Anobile et al., 2021a), with such advantage correlating with their calculation skills (Ciccione and Dehaene, 2020), no groupitizing effect occurs in pre-schoolers (Starkey and McCandliss, 2014). Furthermore, a recent fMRI study showed that perception of grouped elements selectively elicited the activation of regions known to be involved in the execution of calculation/arithmetical fact retrieval, such as bilateral fronto-parietal network and angular gyrus (Maldonado Moscoso et al., 2022).

A still open question is at what stage of the numerosity perception hierarchy, the groupitizing phenomenon emerges. Previous event-related potential (ERP) studies showed that numerosities perception in the subitizing and estimation ranges are two quite different processes (Libertus et al., 2007; Hyde and Spelke, 2009, 2011; Fornaciai and Park, 2017). For example, in an experiment involving a numerical comparison task with symbolic (Arabic numerals) and non-symbolic (arrays of dots) stimuli, participants had to indicate whether stimuli in the subitizing range (1–4) or in the estimation range (6–9) were larger or smaller than the standard stimulus equal to 5 (Libertus et al., 2007). For non-symbolic stimuli, the amplitude of the N1 component increased with the absolute numerical values of the stimuli (up to 6) regardless the numerical distance from the standard stimulus while, in a second experiment, no difference in the N1 component was found for larger numerical sets spanning from 8 to 30 items. Similarly, using a passive viewing task, Fornaciai and Park (2017) found that the amplitude of an early negative component was gradually modulated for arrays containing items within the subitizing range (the smaller the quantity, the smaller the negative-polarity deflection). However, such modulation was absent for larger numerosities (100–400 dots) to suggest different neural activities for quantities that fall within or outside the subitizing range. Hyde and Spelke (2009, 2012) conducted two studies with an adaptation paradigm in which participants passively viewed dot arrays in the subitizing (1–3) or the estimation (8–24) ranges. Participants sequentially viewed adaptor and occasional test stimuli presenting the same or a different number. The results showed that the N1 component was modulated in peak latency by the absolute number in both ranges with latencies shortening as numerosity increased. However, while in the subitizing range the increase in numerosity was mirrored by an increase of the N1 amplitude, the same did not hold for numerosities in the estimation regime. In contrast, while the amplitude of a later component (P2p) was found to positively correlate with the ratio difference between the adaptor and the test in the estimation regime, the same did not occur for subitizing.

The article "EEG signature of grouping strategies in numerosity perception" was published in 2023. Journal: Front Neurosci.

Overall, these results show that processing of large and small numbers could entail different mechanisms involving the activity of partially distinct neural signatures. According to Hyde and Spelke (2009, 2012), the modulation of the N1 component, in both latency and amplitude, found with very small numbers would reflect the distribution of attention in space and object tracking mechanisms. In line with this view, studies that manipulated the distribution of spatial attention have reported a similar modulation of the N1 component (Hillyard et al., 1990, 1998; Hillyard and Anllo-Vento, 1998; Luck, 2005). Here we aim at investigating whether groupitizing drives specific electrophysiological responses, reflecting the interaction of subitizing mechanisms when the overall numerosity is within the estimation range but elements are grouped into small ensembles. To this aim, we measured ERP responses while participants performed a numerosity estimation task on stimuli within the subitizing range (3 and 4 items) or within the estimation range (6 and 8 items). In the latter case, the stimuli could be either organized into small clusters (grouped condition) or being randomly scattered (ungrouped condition). In the grouped condition, stimuli were divided into subgroups within the range of subitizing (3 and 4 subgroups). If groupitizing affects the processing of the number of elements in a scene, we expect to find differences in the response to stimuli in the estimation range depending on the spatial arrangement (grouped or ungrouped). More specifically, we expect to find a signature of the subitizing system (i.e., similar ERP components) whenever stimuli in the estimation range are grouped to form subitizable clusters. Finally, to evaluate the relative weight of the subitizing and estimation systems in the grouped condition, we separately analyzed ERP patterns for trials in which the number of subgroups (in the subitizing range) covaried with the total numerosity of items (in the estimation range; congruent condition) and those in which the number of subgroups and the total numerosity were inversely related (incongruent condition).

## Materials and methods

### Power analysis

Sample size was calculated using a Power analysis (G*Power software, version 3.1). The main goal of the current experiment was to explore the differences in the event related potentials between quantities grouped or randomly sparse. For this reason, the Power analysis calculated the sample size needed to reliably detect a significant difference across small and medium numerosities (1–10) in N1 and P2p components of the ERPs. The effect size was estimated from previous studies that measured ERPs in a numerosity estimation task (Ester et al., 2012; Mazza et al., 2013). With an *⍺* = 0.05 and a Power of 0.9, the analyses suggested a required sample size of 21 participants.

### Participants

Twenty-seven participants took part in the study. Five participants were excluded from analysis due to poor quality of the EEG signal. The final sample comprised 22 participants (mean age: 23.09 years; standard deviation: 3.34; 9 males, two authors) with normal or corrected to normal visual acuity. The research was approved by the ethics committee (Commissione per l’Etica della Ricerca, University of Florence, July 7, 2020, n. 111). The research was performed in accordance with Declaration of Helsinki and informed consent was obtained from all participants prior to each experiment.

The article "EEG signature of grouping strategies in numerosity perception" was published in 2023. Journal: Front Neurosci.

### Materials and procedure

Participants sat 57 cm away from a 23″ screen monitor (resolution 1920 × 1080 pixel; refresh rate 60 Hz), in a quiet and dimly lit room, and estimated the numerosity of a centrally presented array of items. In different sessions participants viewed arrays of 3 and 4 items (targeting the subitizing system) or 6 and 8 items (targeting the estimation range, see Figure 1). Sessions testing the estimation range entails arrays of 6 and 8 items that were either randomly arranged or spatially segregated in groups (3 or 4 subgroups, see Figure 1A).

**Figure 1:** Stimuli configuration and overview of the experimental design. **(A)** Examples of stimulus configurations in estimation and subitizing ranges. **(B)** Participants performed eight sessions estimating quantities in the estimation range, each comprising four blocks with grouped (G) and ungrouped (U) stimuli alternated and one session estimating quantities within the subitizing range. **(C)** Example of the time course of the stimuli.

Each trial started with a white central fixation point that remained on screen for the entire experiment. After 1 s an array of items was centrally displayed for 200 ms, followed by a blank screen and participants had to verbally report the numerosity of the array (Figure 1C). The experimenter pressed the spacebar as soon as the response was spelled out and entered the response on the numeric keypad. Participants were asked to respond as quickly and accurately as possible.

Each participant completed 9 sessions: 1 session of 128 trials for stimuli in the subitizing range and 8 sessions of 64 trials each for stimuli in the estimation range. In half of the trials of the estimation range, stimuli were spatially grouped (grouped condition) while in the other half they were pseudo-randomly scattered in space (ungrouped condition) and the two conditions alternated across the session (Figure 1B). In order to dissociate changes in the overall numerosity from changes in the number of subgroups, in the grouped condition half of the trials displayed the overall numerosity as parsed in a congruent number of subgroups (6 items arranged in 3 groups and 8 items arranged in 4 groups), while in the other half of the trials these factors were inversely related (6 items arranged in 4 groups and 8 items arranged in 3 groups, to have the higher numerosity entailed in fewer groups and viceversa). Each participant performed a total of 640 trials. Stimuli were generated and presented with PsychToolbox 3.0.16 routines (Brainard, 1997; Kleiner et al., 2007) for Matlab (Ver. R2018b 9.5, The Mathworks, Inc.).^1^

The article "EEG signature of grouping strategies in numerosity perception" was published in 2023. Journal: Front Neurosci.

### Stimuli

#### Estimation range

Stimuli were arrays of 6 or 8 white squares (0.4 deg × 0.4 deg) with black borders, with overall luminance matched to the grey background, with a total surface area of 0.96 deg^2^ for 6 items and of 1.28 deg^2^ for 8 items. Squares could not overlap and were constrained to fall within a central 6.5 deg × 6.5 deg virtual square area (total field area), and a convex hull of 19.3 ± 0.8 deg^2^. In the ungrouped condition, the position of each square was randomly selected from 106 possible locations within the central virtual square area. In the spatially grouped condition, each numerosity was arranged into 3 or 4 subgroups, each comprising a variable number of items, resulting in the following configurations: 2–2-2, 3–1-2, 3–1–1-1, 2–2–1-1, 3–3-2, 4–2-2, 2–2–2-2, 3–2–2-1.

#### Subitizing range

Stimuli comprised arrays of 3 or 4 white squares with black borders displaced in the same locations and covering the same area of grouped stimuli in the estimation range (Figure 1). Both 3 and 4 squares covered a total field area of 6.5 deg × 6.5 deg, with a convex hull of 19.3 ± 0.8 deg^2^ and a total surface area equal to 6 items (0.96 deg^2^) for half trials and equal to 8 items (1.28 deg^2^) for half trials.

### EEG recording and preprocessing

EEG signal was recorded throughout all the experiment with a g.Nautilus Multi-Purpose system (gTEC, Austria) from 30 g.SCARABEO active gel-based electrodes (FP1, FP2, F7, F3, Fz, F4, F8, FC5, FC1, FC2, FC6, C3, Cz, C4, CP5, CP1, CP2, CP6, P7, P3, Pz, P4, P8, PO7, PO3, POz, PO4, PO8, O1, O2). The signal was referenced online to the right earlobe and the ground electrode was placed on AFz. Electrooculogram (EOG) were also collected to monitor blinking and eye movements from the outer canthus of both eyes. Impedances were kept below 30 kΩ. The signal was recorded with a high-pass filter of 0.01 Hz and digitized at a sampling rate of 500 Hz. Pre-processing was carried out using custom routines in Matlab (Ver. R2021b 9.11 The Mathworks, Natick, MA, United States) and EEGLAB v14.1.2 (Delorme and Makeig, 2004).

The signal was filtered offline with a Hamming-windowed sinc FIR filter, between 1 and 40 Hz. We identified bad channels by visual inspection and we removed and interpolated electrodes with a spherical interpolation method (average interpolated channels: 6.8%). Data from all electrodes were re-referenced offline to the average of all electrodes. Epochs (from 500 ms before the stimulus to 1,000 ms after the presentation of the stimulus) were extracted from the continuous signal and those contaminated by excessive muscular artifacts were excluded by visual inspection. In total, 4.5% of epochs were excluded. Eye-blinks and residual anterior muscle artifacts were removed by applying Infomax Independent Component Analysis (ICA), (average removed ICs: 7.9). Finally, pre-stimulus baseline was removed (−200 ms to 0).

The article "EEG signature of grouping strategies in numerosity perception" was published in 2023. Journal: Front Neurosci.

### Data analysis

#### Behavioural

Behavioural data were separately analysed for each participant. We first calculated the accuracy of numerical estimation (i.e., the average perceived numerosity) and the precision (as the responses’ standard deviation), separately for each numerosity and condition. The groupitizing effect was indexed in terms of precision by normalizing the standard deviation of the responses distribution by the average perceived numerosity to achieve Weber fraction (Wf), a dimensionless index of precision. Weber fraction was defined as:


(1) $$Wf=\frac{\sigma }{N}$$

where *N* is the average response to a specific numerosity and σ the standard deviation of responses distribution. Higher Weber fraction values indicate lower levels of precision in numerosity estimates.

Behavioural data of the numerosity estimation range were analysed with a Repeated Measures ANOVA and Bonferroni corrected post-hoc t-tests (with *p*-values corrected for multiple comparisons reported as p_bonf_). Effect sizes (*η*^2^) were also reported where appropriate. Statistical analyses were performed using JASP (version 0.16.1, The JASP Team 2022).^2^

#### Event related potentials

Event-related potentials were analysed by quantifying latency and amplitude modulation of each component of interest (N1, P2p) throughout the different experimental conditions. For each component of interest, we merged ERP responses across the different experimental conditions, extracted the topographical activation map corresponding to the peak of the component (N1 or P2p) and then selected cluster of electrodes showing maximal (positive or negative) amplitude values. This procedure led to select electrodes PO3, PO4, PO7, PO8, POz, O1 and O2 in the N1 time range and electrodes PO3, PO4, POz, P3, P4 and Pz in the P2p time range. To assess the peak latency of N1, we used the percent-area latency, a measure that is robust to high-frequency noise and that detects the time point in a specific time window when the component has reached a predefined percentage of its area under the curve (50%, Liesefeld, 2018). The latency estimates were extracted from data, using the MATLAB (The Mathworks, Natick, MA, United States) function latency.m (Liesefeld, 2018). To estimate the amplitude of N1, we calculated the average value in a temporal range of activity (40 ms) around the individual peak latency. With regard to the P2p component, since it was impossible to calculate the peak latency of the component (see Results section below for further details), we estimated the amplitude by averaging the values in a *a-priori* temporal window (210–250 ms), in line with the typical values reported in literature (Libertus et al., 2007).

The article "EEG signature of grouping strategies in numerosity perception" was published in 2023. Journal: Front Neurosci.

ERP data were analysed by parametric Paired-Sample *T*-tests (t-Student, t, two tails) and Repeated measures ANOVAs. When appropriate we performed Bonferroni corrected *post-hoc t*-tests (p_bonf_). Effect sizes were reported as *η*^2^ or Cohen’s *d*.

## Results

### Behavioural results

We first investigated the effect of grouping on the accuracy of perceived numerosity. In line with previous findings (Anobile et al., 2020), we found no differences in perceived numerosity between grouped and ungrouped conditions, both with 6 (grouped condition: mean: 6.35, standard deviation: 0.39; ungrouped condition: mean: 6.34, standard deviation: 0.35) and 8 (grouped condition: mean: 7.96, standard deviation: 0.55; ungrouped condition: mean: 8.00, standard deviation: 0.61) items. To statistically test differences across conditions, we performed a Repeated measure ANOVA with numerosity (2 levels: 6 or 8 items) and spatial arrangement (2 levels, ungrouped or grouped) as factors. Results revealed a significant main effect of numerosity [*F*(1,21) = 452.1, *p* < 0.001, η^2^ = 0.947], but no significant effect of spatial arrangement [F(1,21) = 0.50, *p* = 0.49, *η*^2^ = 0.0001] and no singnificant interactions between factors [F(1,21) = 3.0, *p* = 0.10, *η*^2^ = 0.0003], showing that grouping did not significantly affect perceived numerosity.

We then evaluated the effect of spatial arrangements on precision to quantify the groupitizing effect. For each numerosity we measured Wfs for spatially grouped and randomly scattered stimuli (Figure 2). The results replicated previous findings (Anobile et al., 2020): Wfs were lower when stimuli were grouped (mean: 0.084, standard deviation: 0.031) compared to when they were ungrouped (mean: 0.090, standard deviation: 0.029).

**Figure 2:** Behavioral results. Average Weber fraction for 6 and 8 items, for both grouped and ungrouped conditions.

A Repeated measures ANOVA, with numerosity (2 levels: 6 or 8 items) and spatial arrangement (2 levels: ungrouped or grouped) as factors, revealed a significant main effect of spatial arrangements [*F*(1,21) = 4.63, *p* = 0.043, *η*^2^ = 0.06] suggesting that the sensory precision of numerical estimates improved when items were grouped. The main effect of numerosity [*F*(1,21) = 0.11, *p* = 0.74, *η*^2^ = 0.003], nor the interaction were statistically significant [*F*(1,21) = 0.001, *p* = 0.97, *η*^2^ < 0.001]. On average, groupitizing improved sensory precision up to about 5%, confirming that groupitizing enhances performance on numerical estimation task.

The article "EEG signature of grouping strategies in numerosity perception" was published in 2023. Journal: Front Neurosci.

### Event related potentials

We focused our analysis on an early negative component (N1) and on a mid-latency posterior component (P2p), as previous studies reported these components to be modulated in response to numerical changes in both the subitizing and estimation range (Libertus et al., 2007; Hyde and Spelke, 2009, 2012; Fornaciai and Park, 2017; Grasso et al., 2022b).

While both latency and amplitude were analysed for the N1 component, we only focused on the amplitude of the P2p component as the peak in the ERP signal was mostly merged with the subsequent P3 component (see Figure 3B). Thus, we determined the P2p amplitude within an *a priori* temporal window (between 210 ms and 250 ms), based on previous studies (Libertus et al., 2007; Grasso et al., 2022b).

**Figure 3:** ERPs responses to stimuli in the subitizing range. ERPs response averaged across electrodes PO3, PO4, PO7, PO8, POz, O1, O2 **(A)** and across electrodes PO3, PO4, POz, P3, P4 and Pz **(B)** for 3 (red curves) and 4 items (blue curves). In panel **(A)**, image insert shows a detail of the N1 component; in panel **(B)**, a detail of the P2p component. N1 latency **(C)**, N1 amplitude **(D)** and P2p amplitude **(E)** in response to low and high numerosities averaged across participants. Error bars represent standard error of the mean corrected for a within-subject design (Cousineau and O’Brien, 2014).

### ERP responses to numerosity in the subitizing range

We first evaluated whether the N1 and P2p components were differently modulated by changes in numerosity within the subitizing range (Figures 3A,B). To this aim we compared the electrophysiological responses to 3 and 4 items, performing paired-sample *t*-tests.

N1 latency (Figure 3C) peaked earlier for 4 (147.2 ± 2.4 ms) compared to 3 (152.5 ± 2.3 ms) items [*t*(21) = 4.09, *p* < 0.001, Cohen’s *d* = 0.87]. On the contrary, N1 and P2p amplitudes (Figures 3D,E) were not modulated by changes in numerosity [N1 component: *t*(21) = 0.98, *p* = 0.340, Cohen’s *d* = 0.21; P2p component: *t*(21) = 0.19, *p* = 0.85, Cohen’s *d* = 0.04]. To summarize, these results clearly revealed that unlike N1 and P2p amplitudes, the analysis of N1 latency was capable to uncover small changes of numerical values within the subitizing range.

### Comparison across spatial arrangements in the estimation range

Next, we investigated whether the N1 and P2p components mirrored changes in numerosity in the estimation range, and most importantly whether they were sensitive to the spatial arrangement of the stimuli (ungrouped and grouped, see Figure 4). To this aim we entered the N1 latency and the N1 and P2p amplitudes in separate repeated measure ANOVAs with numerosity (2 levels: 6 and 8 items) and spatial arrangement (2 levels: grouped and ungrouped) as factors.

The article "EEG signature of grouping strategies in numerosity perception" was published in 2023. Journal: Front Neurosci.

**Figure 4:** N1 latency **(A)**, N1 amplitude **(B)** and P2p amplitude **(C)** in response to 6 and 8 items separately for the ungrouped (red circles) and grouped condition (purple squares) averaged across participants. Error bars represent standard error of the mean corrected for a within-subject design (Cousineau and O’Brien, 2014).

The main effect of numerosity was significant for N1 latency [*F*(1,21) = 28.39, *p* < 0.001, *η*^2^ = 0.17], with 8 items (152.7 ± 2.0 ms) eliciting an earlier N1 peak as compared to 6 items (154.0 ± 1.9 ms) to indicate that N1 latency is tuned to numerosity of the set also in the estimation range (Figure 4A). On the contrary, the main effect of numerosity was not significant for the N1 amplitude [*F*(1, 21) = 2.16, *p* = 0.16, *η*^2^ = 0.03; Figure 4B], to suggest that N1 latency is more sensitive to changes in numerical values than N1 amplitude. The factor of spatial arrangement was not significant neither considering N1 latency [*F*(1,21) = 2.10, *p* = 0.16, *η*^2^ = 0.04] nor its amplitude [*F*(1,21) = 3.54, *p* = 0.07, *η*^2^ = 0.07]. Also the interaction between the factors numerosity and spatial arrangement was not significant neither when N1 latency [*F*(1,21) = 0.66, *p* = 0.43, *η*^2^ = 0.008] nor when amplitude [*F*(1,21) = 0.003, *p* = 0.96, *η*^2^ < 0.0001] were taken into account, suggesting that grouped and ungrouped stimuli elicited similar N1 components in response to numerosity changes.

In contrast, the amplitude of the P2p component (Figure 4C) showed both, a main effect of numerosity [*F*(1,21) = 6.77, *p* = 0.02, *η*^2^ = 0.09] and a main effect of spatial arrangement [*F*(1,21) = 6.66, *p* = 0.02, *η*^2^ = 0.10]. P2p amplitude was higher for 8 (1.74 ± 0.36 μV) compared to 6 (1.52 ± 0.36 μV) items and for grouped (1.74 ± 0.36 μV) compared to ungrouped (1.52 ± 0.36 μV) stimuli. The interaction between these factors was not significant [*F*(1,21) = 0.28, *p* = 0.60, *η*^2^ = 0.003].

Overall, these results suggest that the P2p amplitude is sensitive to both the total numerosity of the array and the spatial arrangement, while the N1 latency is mostly sensitive to the total numerosity.

However, since our previous analysis showed that the N1 latency was strongly modulated by numerosities in the range of subitizing, we next asked whether it also reflected the number of subgroups (also in the subitizing range) in addition to total numerosity. To this aim, within the grouped condition we separately analysed trials in which the total numerosity and the number of subgroups varied congruently (congruent condition, i.e., 6 items grouped into 3 clusters and 8 items grouped into 4 clusters, Figure 5A) from those in which these two factors were inversely related (incongruent condition, i.e., 6 items grouped into 4 clusters and 8 items grouped into 3 clusters, Figure 5B).

The article "EEG signature of grouping strategies in numerosity perception" was published in 2023. Journal: Front Neurosci.

**Figure 5:** ERPs responses to grouped stimuli in the estimation range. ERPs response averaged across electrodes PO3, PO4, PO7, PO8, POz, O1, O2 for 6 (orange) and 8 (blue) items in **(A)** the congruent condition (6 items divided in 4 subgroups and 8 items divided in 4 subgroups) and in **(B)** the incongruent condition (6 items divided in 4 subgroups and 8 items divided in 3 subgroups). Image inserts in panels **(A,B)** show the peak latency of the N1 component. N1 latency **(C)**, N1 amplitude **(D)** and P2p amplitude **(E)** in response to 6 and 8 items separately for the ungrouped (red circles), grouped- Congruent (N6 grouped into 3 clusters and N8 grouped into 4 clusters; blue squares) and grouped- Incongruent (N6 grouped into 4 clusters and N8 grouped into 3 clusters; green squares) condition averaged across participants. Error bars represent standard error of the mean corrected for a within-subject design (Cousineau and O’Brien, 2014).

In the congruent trials (Figure 5C, blue line), N1 latency was much more strongly modulated by numerosity compared to the ungrouped condition (Figure 5C, red hatched line), with higher numerosities (both of subgroups and total) eliciting shorter latencies for higher numbers, similarly to what observed for the subitizing range in our previous analysis. Most strikingly, in the incongruent trials (Figure 5C, green line), the N1 latency appeared to be driven by the number of subgroups (within the subitizing range) and not by total numerosity.

Repeated measures ANOVA, with numerosity (2 levels: 6 or 8 items) and congruency (2 levels: congruent and incongruent conditions) as factors, confirmed the significant interaction for the latency [*F*(1,21) = 54.02, *p* < 0.001, *η*^2^ = 0.51]. *Post-hoc t*-tests showed that, when the number of subgroups congruently covaried with the total number of items, the latency of the N1 component was shorter for 8 compared to 6 items [*t*(21) = 7.71, *p*_bonf_ < 0.001, Cohen’s *d* = 0.52; Figure 5A]. However, when the number of subgroups were inversely related to the total numerosity, the latency decreased with the number of subgroups being shorter for 6 items grouped in 4 ensembles compared to 8 items grouped in 3 ensembles [*t*(21) = −4.38, *p*_bonf_ < 0.001, Cohen’s *d* = −0.29; Figure 5B]. Overall, this result suggests that the number of subgroups more than the total numerosity of items modulated the N1 latency when these factors are at odds to each other. On the other hand, when the number of subgroups and the total numerosities were congruent, they probably enhanced each other eliciting stronger modulations of the N1 latency compared to the ungrouped condition.

The article "EEG signature of grouping strategies in numerosity perception" was published in 2023. Journal: Front Neurosci.

Following the same logic, we next performed the same analysis on the amplitudes of the N1 and P2p components. A similar trend to that observed for the N1 latency was observed also for the N1 amplitude (Figure 5D): the N1 amplitude decreased with both the number of subgroups and total numerosity in the congruent trials, while it was primarily modulated by the number of subgroups in the incongruent trials. This effect was however much weaker compared to what observed in latency and despite the interaction between numerosity and congruency was significant [*F*(1,21) = 5.24, *p* = 0.033, *η*^2^ = 0.09], none of the post-hoc reached significance.

The amplitude of the P2p component (Figure 5E) was modulated by total numerosity (increase in amplitude for higher numerosity), regardless of congruency (and hence of the number of subgroups). The Repeated measures ANOVA confirmed a significant main effect of numerosity [*F*(1, 21) = 5.21, *p* = 0.033, *η*^2^ = 0.11] and no effect of congruency [*F*(1, 21) = 1.75, *p* = 0.20, *η*^2^ = 0.01] nor interaction between factors [*F*(1, 21) = 2.80, *p* = 0.11, *η*^2^ = 0.04], suggesting that the P2p component responds to the total numerosity of items.

Taken together these results suggest that the ERP responses to arrays of different numerosities change when grouping cues are available. Interestingly, while the P2p amplitude was higher for grouped compared to ungrouped numerosities irrespective of the congruency between the total numerosity and number of subgroups, the N1 latency reflected the numerosity in the set when stimuli were randomly distributed, but when grouping cues were available, it primarily reflected the number of groups even when it was at odds with the total numerosity of the array (see Table 1 for a summary of the results).

**Table 1:** Summary of the results in the estimation range.

Condition	N1 Latency		N1 Amplitude		P2p Amplitude	
	*N* = 6	*N* = 8	*N* = 6	*N* = 8	*N* = 6	*N* = 8
Ungrouped	153.8 ± 2.0 ms	152.3 ± 2.1 ms*	−5.4 ± 0.5 μV	−5.5 ± 0.5 μV	1.4 ± 0.4 μV	1.6 ± 0.3 μV
Congruent	156.0 ± 1.8 ms	151.4 ± 1.9 ms*	−5.1 ± 0.5 μV	−5.5 ± 0.6 μV	1.6 ± 0.3 μV	2.0 ± 0.4 μV
Incongruent	152.5 ± 2.1 ms	155.1 ± 1.8 ms*	−5.3 ± 0.5 μV	−5.2 ± 0.5 μV	1.6 ± 0.4 μV	1.8 ± 0.4 μV

The table shows the N1 latency, N1 amplitude and P2p amplitude averaged across participants for the different numerosities and conditions (Ungrouped, Congruent, and Incongruent). “Ungrouped” refers to the condition in which items were randomly displayed, “Congruent” to the condition in which the number of groups increased congruently with number of items (i.e., 6 items arranged into 3 groups and 8 items arranged into 4 groups) while “Incongruent” indicates the condition in which the increase in the number of groups paralleled a decrease in the number of items (i.e., 6 items arranged into 4 groups and 8 items arranged into 3 groups). Asterisks depicts significant comparisons between N6 and N8 (i.e., *p* < 0.05). Errors represent standard error of the mean corrected for a within-subject design (Cousineau and O’Brien, 2014).

The article "EEG signature of grouping strategies in numerosity perception" was published in 2023. Journal: Front Neurosci.

Since the number of subgroups was in the subitizing range, we next evaluated whether the responses to the number of subgroups was more comparable to those to individual items in the subitizing range or to those to ungrouped items in the estimation range. To this aim we calculated the N1 latency difference for stimuli in the subitizing range and compared it to the difference in N1 latencies in the estimation range when numerosities were ungrouped or parsed in the corresponding number of subgroups (congruent trials). We used congruent trials because this was the only condition allowing us to simultaneously compare responses to stimuli with the same number of items/groups (subitizing vs. grouped trials) and with the same number of overall items (ungrouped vs. grouped trials.).

To evaluate whether the difference in N1 latency elicited by numerosity changes in the subitizing range was more similar to that in the estimation range for randomly scattered or grouped stimuli, we calculated the N1 latency differences for each participant, by subtracting the latency in response to the higher from the lower numerosity (Figure 6). We entered these values in a Repeated measure ANOVA with condition as factor (subitizing, ungrouped and congruent grouped trials). The significant main effect of condition [*F*(42,2) = 5.59, *p* = 0.007, *η*^2^ = 0.21] and post-hoc t-tests showed a significant latency difference between the subitizing and estimation ranges but only when items were ungrouped [*t*(21) = 3.13, *p*_bonf_ = 0.009, Cohens’*d* = 0.94], while this difference was not significant for the congruent trials [*t*(21) = 0.60, *p*_bonf_ = 1.00, Cohens’*d* = 0.18]. Moreover, the difference between grouped and ungrouped stimuli was significant [*t*(21) = 2.54, *p*_bonf_ = 0.045, Cohens’*d* = −0.77], showing that the N1 latency differences between 8 and 6 items depends on the spatial arrangement. Overall, these results suggest that the latency difference across numerosities for grouped stimuli in the estimation range is comparable to the one observed for stimuli in the subitizing range.

The article "EEG signature of grouping strategies in numerosity perception" was published in 2023. Journal: Front Neurosci.

**Figure 6:** N1 latency differences. The bar graph shows the N1 latency differences (high – lower numerosity, in ms) averaged across participants in response to stimuli in the subitizing (grey), and in the estimation range for ungrouped (red) and congruent grouped (green) stimuli (* = *p* < 0.05; ** = *p* < 0.01). Error bars represent standard error of the mean corrected for a within-subject design (Cousineau and O’Brien, 2014).

## Discussion

This study explored the electrophysiological correlates of “groupitizing.” We measured ERP responses while participants were involved in a numerosity estimation task with quantities either falling in the subitizing or in the estimation ranges. In the latter case, we contrasted ERP responses to items randomly scattered in space or clustered in subgroups. The activation of the subitizing system is thought to be fundamental for the groupitizing phenomenon (Maldonado Moscoso et al., 2020), therefore in the current study we aimed at identifying an electrophysiological signature of the subitizing system when processing grouped arrays of items of larger numerosities falling in the estimation range.

A previous study showed that the N1 latency is modulated by changes in numerosity across both the subitizing and the estimation range (Hyde and Spelke, 2009). Here we confirmed this result, by showing that, in both ranges, as numerosity increased (from 3 to 4 items in the subitizing range and from 6 to 8 items in the estimation range) the N1 peaked earlier. In the estimation range, this held true not only for the ungrouped, but also for the grouped condition. Nevertheless, we also found that N1 latencies in response to grouped stimuli depended on the congruency between the total numerosity and the number of subgroups which determined the direction of the latency modulation (either increasing or decreasing) with total numerosity. Of note, this opposed pattern is likely to explain why we were not able to highlight differences between grouped and ungrouped stimuli when the two conditions (congruent and incongruent) were kept together. We here investigated whether changes in electrophysiological responses reflected changes in total numerosity and/or changes in the number of groups when these two factors were varied either congruently or incongruently. The rationale was: if groupitizing is based on the recruitment of the subitizing system, the electrophysiological response to grouped stimuli should also reflect the number of subgroups when their numerosity falls in the subitizing range in addition to the total numerosity (falling in the estimation range). This prediction was supported by multiple evidence. First, when the number of subgroups congruently varied with the total numerosity (congruent trials), the latency difference between 6 and 8 items was much amplified compared to when the same numerosities were ungrouped, resembling the latency modulation occurring when processing numerical changes of the same ratio in the subitizing range (3 vs. 4 items). This similarity was quantitatively verified by comparing the latency difference across numerosities in the subitizing and estimation ranges, with both ungrouped and grouped items: the latency difference between high and low numerosities elicited by grouped stimuli was different from the one elicited by the very same numerosities (6 vs. 8) when items were randomly arranged in space, while it did not differ from the one elicited by stimuli in the subitizing range (3 vs. 4, corresponding to the number of subgroups in the grouped stimuli). This suggests that the presence of subgroups (within the subitizing range) boosted the latency difference between numerosities in response to the (congruent) grouped trials in the estimation range, reminiscent of the latency difference between 3 and 4 items. Second, in the incongruent trials, in which the number of subgroups and the total numerosity were inversely related, the number of subgroups rather than the overall numerosity modulated the N1 latency. Specifically, six elements grouped into four clusters elicited shorter N1 latency as compared to eight elements grouped into three clusters which is opposed to what was expected to occur if the total number of elements modulated the N1 latency. Most strikingly, based on the N1 latency we were nevertheless able to discriminate between numerosities in the subitizing range (3 and 4 items) from the number of subgroups (3 and 4 clusters with total numerosity of items in the estimation range): the N1 latency in response to grouped stimuli was within the typical latency range of estimation (around 153 ms) and did not approach the latency range of subitizing (around 149 ms). Overall, these results suggest that the N1 latency was probably modulated by both the subitizing and the estimation systems in response to grouped numerosities: the N1 latency modulation for numerosities in the congruent trials was mainly driven by the number of subgroups, yet remaining within the latency range observed for quantities in the estimation range.

The article "EEG signature of grouping strategies in numerosity perception" was published in 2023. Journal: Front Neurosci.

It is important to note that the results in our experiment are unlikely explained by low-level features of the stimuli (e.g., total field area, total surface area, convex hull), as numerosities in the subitizing range were matched on average luminance, total field area and convex hull and those in the estimation range had same average convex hull and total field area. Stimuli in the estimation range differed in terms of luminance (8 items had higher luminance than 6 items). However, the N1 latency modulation to the same numerosities reversed in the congruent compared to the incongruent conditions, suggesting that N1 latency was not driven by luminance (Johannes et al., 1995).

In the current study we observed that the N1 amplitude decreased with numerosity both in the subitizing and in the estimation ranges, although this decrement was not statistically significant. For numerosities in the subitizing range, this result is in contrast with previous findings (Libertus et al., 2007; Hyde and Spelke, 2009, 2012; Fornaciai and Park, 2017). However, this difference is likely attributable to the ratio between numerosities used here (very small, 1.33) compared to those previously used by others (1.5, 2, 3 or 4, Libertus et al., 2007; Hyde and Spelke, 2009; Fornaciai and Park, 2017). Similarly to N1 latency, also N1 amplitude did not significantly discriminate between spatial configurations for grouped stimuli in the estimation range. However, differently from the N1 latency, the N1 amplitude showed a much weaker modulation with congruency between total numerosity and number of subgroups, albeit showing a similar tendency.

Overall, the current study identifies in the N1 component (although most clearly in its latency), the electrophysiological signature of the subitizing system during groupitizing, reinforcing the hypothesis that this phenomenon leverages on the spontaneous capacity to subitize and that its influence is located at the early individuation stage (Mazza and Caramazza, 2012).

Previous ERP studies ascribed the modulation of the N1 component, mostly its amplitude, to several cognitive functions including visuo-spatial attention [see reviews by Mangun (1995), Hillyard and Anllo-Vento (1998)] and visual discrimination processes (Mangun and Hillyard, 1991; Martínez et al., 1999; Vogel and Luck, 2000; Grasso et al., 2016). Regarding the modulation of the N1 latency, previous studies showed that it varied according to the amount of effort needed to solve a task, with later latency elicited by more complex tasks (Callaway and Halliday, 1982; Fort et al., 2005).

The modulation of the N1 component evoked by numerosity of stimuli observed in the current study might therefore reflect a perceptual mechanism that extracts the information of the overall number of elements and guarantees the distribution and the maintenance of attention to item locations in the visual field (Hyde and Spelke, 2012; Mazza et al., 2013; Mazza and Caramazza, 2015). This would be in line with evidence showing that the subitizing system relies on cognitive resources such as attention and working memory (Burr et al., 2010; Melcher and Piazza, 2011; Piazza et al., 2011). These studies found that subitizing capacity is correlated with visual–spatial working memory ability suggesting that both subitizing and visuo-spatial working memory share a mechanism which simultaneously tracks multiple objects in parallel and explicitly represents their spatial positions (Piazza et al., 2011).

The article "EEG signature of grouping strategies in numerosity perception" was published in 2023. Journal: Front Neurosci.

Previous studies found that the amplitude of a positive mid-latency component (i.e., P2p) scales with the total numerosity of the stimuli in the estimation range whether or not this difference is real (Park et al., 2016; Fornaciai and Park, 2017) or only perceived (Grasso et al., 2022b). Here we replicated these findings by reporting lower P2p amplitudes for 6 compared to 8 items (although not for 3 versus 4 items, again probably due to the small ratio difference between numerosities as discussed above). Most interestingly, we found that the P2p amplitude was modulated by the spatial arrangement of the stimuli, with grouped stimuli eliciting higher P2p amplitudes. This was observed for both congruent and incongruent trials, suggesting that the P2p amplitude code for the total numerosity irrespective of the number of subgroups. It has been previously showed that the P2p component is affected by cognitive processes such as spatial attention and working memory (Anllo-Vento and Hillyard, 1996; Mecklinger and Müller, 1996) with higher amplitudes reflecting higher cognitive load (Freunberger et al., 2007; Grasso et al., 2020, 2021c). In this view, the larger P2p amplitudes observed in the grouped condition could reflect the involvement of cognitive resources necessary to parse stimuli both in terms of subgroups and in terms of elements within each subgroup, a process that likely requires a larger recruitment of visuo-spatial working memory compared to the ungrouped condition. Nevertheless, the lack of a dissociation between the congruent and the incongruent conditions seems to suggest that this component is not very sensitive to code changes in the number of subgroups.

In conclusions, in the current study we reported the first evidence of the electrophysiological markers subtending the phenomenon of groupitizing. We showed that the N1 component is particularly sensitive to code both the total number of elements and the number of subgroups in which elements are parsed suggesting that this component could be crucially implicated in the emergence of groupitizing advantage. Conversely, the P2p component seems to be much more bounded to the number of elements and to be mostly blind to the number of subgroups in which elements are parsed.

The article "EEG signature of grouping strategies in numerosity perception" was published in 2023. Journal: Front Neurosci.

## Data availability statement

Behavioral and EEG results are publicly available at the following address: https://doi.org/10.5281/zenodo.7913116.

## Ethics statement

The studies involving human participants were reviewed and approved by the Commissione per l’Etica della Ricerca, University of Florence, July 7, 2020, n. 111. The patients/participants provided their written informed consent to participate in this study.

## Author contributions

PM, PG, and EC contributed to conception and design of the study. CC and PM collected the data. CC performed the statistical analyses and wrote the first draft of the manuscript. RA and EC supervised the project. All authors contributed to manuscript revision, read, and approved the submitted version.

## Funding

This research was funded from the European Union (EU) and Horizon 2020—grant agreement no. 832813—ERC Advanced “Spatio-temporal mechanisms of generative perception—GenPercept,” from the Italian Ministry of Education, University, Research under the PRIN2017 programme (grant no. 2017XBJN4F—“EnvironMag” and grant no. 2017SBCPZY—“Temporal context in perception: serial dependence and rhythmic oscillations”), and with the contribution of the researcher Paolo Antonino Grasso with a research contract co-funded by the European Union - PON Research and Innovation 2014–2020 in accordance with Article 24, paragraph 3a, of Law No. 240 of December 30, 2010, as amended, and Ministerial Decree No. 1062 of August 10, 2021.

## Conflict of interest

The authors declare that the research was conducted in the absence of any commercial or financial relationships that could be construed as a potential conflict of interest.

## Publisher’s note

All claims expressed in this article are solely those of the authors and do not necessarily represent those of their affiliated organizations, or those of the publisher, the editors and the reviewers. Any product that may be evaluated in this article, or claim that may be made by its manufacturer, is not guaranteed or endorsed by the publisher.

## Footnotes

^1^ http://mathworks.com

^2^ https://jasp-stats.org/
